# 24-Hour Rhythms of DNA Methylation and Their Relation with Rhythms of RNA Expression in the Human Dorsolateral Prefrontal Cortex

**DOI:** 10.1371/journal.pgen.1004792

**Published:** 2014-11-06

**Authors:** Andrew S. P. Lim, Gyan P. Srivastava, Lei Yu, Lori B. Chibnik, Jishu Xu, Aron S. Buchman, Julie A. Schneider, Amanda J. Myers, David A. Bennett, Philip L. De Jager

**Affiliations:** 1 Division of Neurology, Department of Medicine, Sunnybrook Health Sciences Centre, University of Toronto, Toronto, Ontario, Canada; 2 Program in Translational Neuropsychiatric Genomics, Department of Neurology, Brigham and Women's Hospital, Harvard Medical School, Boston, Massachusetts, United States of America; 3 Program in Medical and Population Genetics, Broad Institute, Cambridge, Massachusetts, United States of America; 4 Rush Alzheimer Disease Center and Department of Neurological Sciences, Rush University, Chicago, Illinois, United States of America; 5 Department of Psychiatry and Behavioral Sciences, Miller School of Medicine, University of Miami, Miami, Florida, United States of America; Roslin Institute and Royal (Dick) School of Veterinary Studies, United Kingdom

## Abstract

Circadian rhythms modulate the biology of many human tissues, including brain tissues, and are driven by a near 24-hour transcriptional feedback loop. These rhythms are paralleled by 24-hour rhythms of large portions of the transcriptome. The role of dynamic DNA methylation in influencing these rhythms is uncertain. While recent work in *Neurospora* suggests that dynamic site-specific circadian rhythms of DNA methylation may play a role in modulating the fungal molecular clock, such rhythms and their relationship to RNA expression have not, to our knowledge, been elucidated in mammalian tissues, including human brain tissues. We hypothesized that 24-hour rhythms of DNA methylation exist in the human brain, and play a role in driving 24-hour rhythms of RNA expression. We analyzed DNA methylation levels in post-mortem human dorsolateral prefrontal cortex samples from 738 subjects. We assessed for 24-hour rhythmicity of 420,132 DNA methylation sites throughout the genome by considering methylation levels as a function of clock time of death and parameterizing these data using cosine functions. We determined global statistical significance by permutation. We then related rhythms of DNA methylation with rhythms of RNA expression determined by RNA sequencing. We found evidence of significant 24-hour rhythmicity of DNA methylation. Regions near transcription start sites were enriched for high-amplitude rhythmic DNA methylation sites, which were in turn time locked to 24-hour rhythms of RNA expression of nearby genes, with the nadir of methylation preceding peak transcript expression by 1–3 hours. Weak ante-mortem rest-activity rhythms were associated with lower amplitude DNA methylation rhythms as were older age and the presence of Alzheimer's disease. These findings support the hypothesis that 24-hour rhythms of DNA methylation, particularly near transcription start sites, may play a role in driving 24-hour rhythms of gene expression in the human dorsolateral prefrontal cortex, and may be affected by age and Alzheimer's disease.

## Author Summary

Circadian rhythms are intrinsic 24-hour biological rhythms that influence many aspects of human biology, including normal and abnormal human brain functions such as cognition and seizures. Circadian rhythms are maintained by a near 24-hour feedback loop mediated by a series of “clock” genes that are similar across species, including humans. However, the specific mechanisms underlying the circadian regulation of gene transcription are unknown. DNA methylation is an epigenetic mechanism that can influence gene expression without changes in DNA sequence. The 24-hour rhythms of DNA methylation are one mechanism contributing to 24-hour rhythms of clock gene expression in fungi. However, this has not been demonstrated in mammals including humans. In this study, we examined levels of DNA methylation at>400,000 sites across the genome in the brains of 738 human subjects and showed significant 24-hour rhythms of DNA methylation. Moreover, we showed that for specific locations of DNA methylation site, these rhythms of methylation were linked to rhythms of gene expression. This is important because it suggests that circadian rhythms of DNA methylation may be an important mechanism underlying circadian rhythms of gene expression in the human brain, and hence circadian rhythms of normal and abnormal brain function.

## Introduction

Circadian rhythms—intrinsic 24-hour biological rhythms—have a major impact on the molecular biology, physiology, and function of many human tissues, including the human brain, where they have an important influence on neurological diseases like dementia, epilepsy, and stroke.

In model organisms, circadian rhythms are generated in neurons of the suprachiasmatic nucleus (SCN) by a transcription-translation feedback cycle involving a set of evolutionarily conserved “clock” genes [1]. Similar clocks are present in other tissues [2], including neocortex. These tissue clocks are entrained by the SCN and drive circadian rhythms of tissue physiology, in part through 24-hour cycles of histone modification and gene expression involving a sizeable subset of the transcriptome [3] that varies from tissue to tissue [4].

Whether circadian rhythms of DNA methylation are important for maintaining or modulating circadian rhythms of gene expression in mammalian tissues is uncertain. Recent work in *Neurospora* suggests that circadian rhythms of DNA methylation may play a role in the fungal molecular clock [5]. Moreover, recent studies demonstrated the importance of non-circadian plastic DNA methylation in mediating the long term effect of light on changes in the period of the intrinsic circadian clock in mice [6], and in mediating the effect of photoperiod on endocrine function in hamsters [7]. However, 24-hour rhythms of promoter region DNA methylation were not found in a study of mouse suprachiasmatic nucleus [6] or in a recent study of mouse liver [8]. To our knowledge, 24-hour rhythms of DNA methylation and their relationship to circadian rhythms of gene expression have not been demonstrated in any mammalian tissue, including human brain.

In fact, there are few studies concerning epigenetic mechanisms influencing circadian rhythms of gene expression in human neocortex. This is an important gap because circadian rhythms exert an important effect on neurological diseases like dementia and epilepsy, as well as on cognition and voluntary human behavior, and the neocortex is central to all of these processes. Understanding and potentially therapeutically manipulating the circadian influence on human neurological diseases and behavior will depend on elucidating their genetic and epigenetic basis in human neocortical tissues. The dorsolateral prefrontal cortex in particular plays a key role in several cognitive domains [9] that show considerable circadian fluctuation, as well as in diseases like schizophrenia [10]. Moreover, significant 24-hour rhythms of gene expression have been demonstrated in human dorsolateral prefrontal cortex [11]. Because the circadian regulation of gene expression varies between tissues and species, there is no perfect substitute for directly studying genetic and epigenetic mechanisms underlying circadian rhythms in human neocortical tissue. However, progress in examining circadian rhythms of epigenetic modification in human neocortex has been limited by difficulties in obtaining large sets of human neocortical specimens at a wide range of circadian times suitable for epigenetic analysis.

The overall aim of this study was to test the hypothesis that 24-hour rhythms of DNA methylation exist in human dorsolateral prefrontal cortex, and play a role in 24-hour rhythms of RNA expression. To do so, we determined DNA methylation levels in post-mortem human dorsolateral prefrontal cortex samples from 738 community-dwelling organ donors at 420,132 autosomal DNA methylation sites across the genome. We considered DNA methylation levels as a function of time of death, parameterized these data using cosine functions, and determined global statistical significance by permutation. We then related 24-hour rhythms of DNA methylation to local gene landmarks, to parallel rhythms of RNA expression determined by RNA sequencing, and to ante-mortem behavioral rhythms measured by actigraphy. We found evidence for widespread 24-hour rhythms of DNA methylation whose timing was closely related to the position of specific DNA methylation sites relative to gene landmarks. Moreover, we found that genomic regions proximate to transcription start site were enriched in high amplitude rhythmic DNA methylation sites, and that the timing of rhythmicity at these sites was time-locked to rhythms of nearby gene expression, with the nadir of methylation preceding peak transcript expression by 1–3 hours. We demonstrated an association between the robustness of ante-mortem rest-activity rhythms and the amplitude of rhythms of DNA methylation. Finally, we identified effects of age, sex, and Alzheimer's disease on the amplitude and phase of rhythms of DNA methylation.

## Results

We analyzed postmortem human neocortical DNA methylation data from 738 individuals participating in 2 longitudinal cohort studies of aging – the Religious Orders Study (ROS) and the Rush Memory and Aging Project (MAP). All ROS and MAP participants are organ donors and hence time of death is well documented. Characteristics of the study subjects are shown in Table 1. DNA methylation levels at 420,132 DNA methylation sites spanning all 22 autosomes was generated using the Illumina Infinium HumanMethylation450 Bead Chip assay (Illumina, San Diego, CA). Prior to further analyses, we accounted for the effects of age, sex, presence/absence of dementia, source cohort, post-mortem interval, and batch effects by regressing the methylation data against these factors and taking the residuals, which were then normalized to the mean and standard deviation of all 738 subjects. These normalized residuals represent the relative methylation at each site adjusted for these covariates, and were used for all further analyses, except where specifically indicated.

**Table 1:** Clinical characteristics of the study subjects.

Characteristic	Mean (SD) or Number (%)
Age at Death (years)	88.0 (6.7)
Female Sex	469 (64%)
Source Cohort	MAP: 340 (46%) ROS: 398 (54%)
Actigraphic Interdaily Stability	0.48 (0.15)
Time of Death (hours)	12:08 (8:11)
Postmortem Interval (hours)	7.5 (5.8)
NIA-Reagan Intermediate/High	446 (60%)

To identify temporal patterns in DNA methylation at each of the sites, we considered DNA methylation as a function of clock time of death, with each subject contributing a single data point to a time series spanning 24 hours. Visual inspection of these data revealed that some sites were clearly rhythmic (Figure 1 A–B) while others were clearly not (Figure 1 C–D).

**Figure 1:** Representative cycling and non-cycling DNA methylation sites. Hash marks indicate means and 95% confidence intervals of the mean. Data are double plotted in 4 hour bins. Red line indicates best-fit cosine curve. (A,B) representative rhythmic DNA methylation sites. (C,D) representative arrhythmic DNA methylation sites. Abbreviations: PVE proportion of variance explained.

Based on visual inspection of these data, and in keeping with prior work examining 24-hour rhythms of gene expression in neocortical tissue [11], we then modeled these data using cosine curves. We parameterized these data using functions of the form M = m+(**β**_1_)*cos(t−**β**_A_)..[Eq1] where m is the mesor (the mean value considering all time points), **β**_1_ is the amplitude of oscillation, **β**_A_ is the timing of the peak, and t is the time of death. We calculated the proportion of variance explained by the fit cosine model at each DNA methylation site (Supporting File 1).

We first carried out a series of analyses to identify global patterns of rhythmicity. To quantify the probability that the observed data could have occurred by chance alone, we performed a series of analyses comparing the observed data to 10,000 permuted null datasets generated by randomly shuffling the times of death in our data while preserving the correlation between DNA methylation sites. We fit cosine curves at each of the 420,132 sites in each null dataset, calculated the proportion of variance at each site explained by the fit cosine curve, and determined the time of the methylation nadir (**β**_A_-**π**). We then carried out four analyses comparing the observed to the 10,000 permuted null datasets: 1) We calculated the mean total proportion of variance collectively explained by the fit cosine curves in each of the 10,000 permuted null datasets and in the observed data, and determined the proportion of null datasets in which this was as large or larger than in the observed data. In none of the 10,000 permuted null datasets was the mean proportion of variance explained by cosine curves greater than in the observed data, indicating that the average rhythmicity of the 420,132 sites is greater than expected by chance alone, and the probability of the observed data being due to chance alone is p<0.0001 (Figure 2A). 2) We repeated the same for the median total proportion of variance explained. As above, in none of the 10,000 permuted null datasets was the median proportion of variance explained by cosine curves greater than in the observed data, indicating p<0.0001 (Figure 2B). 3) We used the Wilcoxon rank-sum test to compare the observed distribution of proportions of variance explained by cosine curves to an empiric null distribution generated by taking the mean of the corresponding vectors from the 10,000 permuted null datasets. The observed distribution was significantly greater than the empiric null distribution (W = 91342066816 p<2.2×10^−16^ by the Wilcoxon rank-sum test). 4) We compared the distribution of methylation nadir times in the observed and permuted null datasets (Figure 2C). As expected, in the permuted null datasets, the methylation nadirs were uniformly distributed. By contrast, the methylation nadirs showed significant non-random clustering in the observed data (H_2_ = 10449.1; p<2.2×10^−16^ by the Rao test for equality of dispersions). Considering these four analyses together, we concluded that the probability of the 24-hour rhythmicity seen in the observed data occurring by chance was exceedingly small.

**Figure 2:** Comparison of observed and permuted null datasets. (A) Mean and (B) Median proportion of methylation variance collectively explained by cosine curves in the 10000 permuted null (open bars) and the observed (red line) datasets, considering all 420,132 sites. In none of the permuted datasets did the mean or median percentage of variance explained exceed that in the observed data, indicating that the probability of the observed data having occurred by chance alone is p<0.0001. (C) Comparison of the timing of the nadirs of methylation at all 420,132 sites in the null (black) and the observed (red) datasets. The nadir times are uniformly distributed in the null datasets. In contrast, the nadir times are significantly non-randomly clustered in the observed data (H_2_ = 10449.1; p<2.2×10^−16^ by the Rao test for equality of dispersions).

DNA methylation is thought to play a role in regulating gene transcription. Therefore, we examined the relationship between the physical position of DNA methylation sites relative to transcription start sites and the observed parameters of rhythmicity such as amplitude and phase (Figure 3). First, we considered all interrogated DNA methylation sites within 20 kb of any GENCODE v14 annotated transcription start site, and plotted the temporal distribution of methylation nadir times in 500 bp bins ranging from −20 kb to +20 kb (Figure 3A). Visual inspection revealed an association between physical position of a DNA methylation site relative to the nearest transcription start site, and the timing of the nadir of methylation, with sites closest to the transcription start site being most likely to reach their methylation nadir in the early morning (∼5:30) while those upstream and downstream being more likely to reach their methylation nadir in the evening (∼20:30). To formally test this, we stratified DNA methylation sites into those between −20 kb and −1 kb of transcription start sites, those between −1 kb and +1 kb of transcription start sites, and those within +1 kb and +20 kb of transcription start sites (Figure 3B). The temporal distributions of methylation nadir times in these three groups differed significantly (H_1_ = 7136.9; p<2.2×10^−16^ by the Rao test for equality of polar direction).

**Figure 3:** The timing and amplitude of DNA methylation at sites near transcription start sites is distinct from other DNA methylation sites. (A) Heat map of the distribution of methylation nadir times as a function of distance from the transcription start site, considering all DNA methylation sites, in 500 bp bins. Each row depicts a one-hour bin of clock time. Red indicates a greater than expected density of methylation nadir times; blue indicates a less than expected density of methylation nadir times. (B) The same data depicted as histograms stratified into three groups: sites between −20 kb and −1 kb relative to the nearest transcription start site, sites between −1 kb and +1 kb of the nearest transcription start site, and sites between +1 kb and +20 kb of the nearest transcription start site. DNA methylation sites near transcription start sites have a tendency to reach their methylation nadir in the early morning, peaking at 5:30, while sites elsewhere are most apt to reach their methylation nadir in the evening, peaking at 20:30 (H_1_ = 7136.9; p<2.2×10^−16^ by the Rao test for equality of polar direction). (C) The proportion of all DNA methylation sites that have a peak to trough difference of more than 10% of the mean methylation level in 500 bp bins relative to the nearest transcription start site. High-amplitude rhythmic DNA methylation sites are enriched in the 1000 kb around transcription start sites (χ^2^ 64712.6, p<2.2×10^−16^).

The higher the amplitude of cycling, the more likely it is to be biologically significant. We therefore examined in more detail the subset of DNA methylation sites with the highest amplitude of cycling. We defined a site as high amplitude if the fit cosine curve had a peak-to-trough amplitude of rhythmicity greater than 10% of the mean value of methylation. We examined the distribution of such high-amplitude sites by dividing the 20 kb upstream and downstream of each transcription start site into 500 bp bins as above, and we determined the proportion of high amplitude DNA methylation sites in each bin. High-amplitude DNA methylation sites were enriched in the 1000 kb around transcription start sites compared to other genomic regions (χ^2^ 64712.6, p<2.2×10^−16^; Figure 3C).

We then repeated the above analyses, except that rather than dividing the genome into bins based on position relative to transcription start sites, we incorporated information about other gene landmarks and divided the genome into 9 bins: regions within 2 kb upstream of transcription start site, in the 5′UTR, in the 1^st^ exon, in the 1^st^ intron, in other exons, in other introns and in the 3′UTR of protein coding transcripts; regions in or within 2 kb upstream of non-protein coding transcripts; and intergenic regions (defined as all other genomic regions). Sites in the 2 kb upstream of transcription start sites, and in the 5′UTR, 1^st^ exon, and 1^st^ intron were most likely to reach their methylation nadir in the early morning, while those in other exons/introns, the 3′UTR, noncoding transcripts, and intergenic regions were most likely to peak in the evening (H1 = 14683.8; p<2.2×10^−16^ by the Rao Test for equality of polar direction; Figure 4A–B). Moreover, the 2 kb upstream of transcription start sites, the 5′UTR, and the 1^st^ exon were relatively enriched in sites with relative high amplitude oscillations as described above (χ^2^ 51250.8, p<2.2×10^−16^; Figure 4C).

**Figure 4:** Sites in gene regions proximate to the transcription start site have a phase and amplitude distinct from other gene regions. (A) Heat map of the distribution of methylation nadir times for DNA methylation sties in various gene regions, considering all GENCODE v14 transcripts. (B) The same data expressed as histograms. Sites in the 2 kb upstream of the nearest transcription start site and in the 5′UTR, 1^st^ exon, and 1^st^ intron are most likely to reach their methylation nadir in the early morning, while those in other exons/introns, the 3′UTR, noncoding transcripts, and intergenic regions are most likely to peak in the evening (H1 = 14683.8; p<2.2×10-16 by the Rao Test for equality of polar direction). (C) The proportion of DNA methylation sites with high amplitude (peak to trough difference of>10% of the mean methylation level) in each gene region. The 2 kb upstream of the TSS, the 5′UTR, and the 1^st^ exon are relatively enriched in sites with high amplitude oscillations (χ^2^ 51250.8, p<2.2×10^−16^).

DNA methylation is hypothesized to play a role in regulating gene transcription. In a subset of 536 participants (Table S1), we generated RNA sequencing data from the same tissue blocks used to generate the DNA methylation data, quantifying the expression level of GENCODE v14 annotated transcripts containing or within 2 kb of high amplitude DNA methylation sites, and detectible in at least 10% of our samples. A total of 69,605 GENCODE transcripts spanning 15,091 genes containing or near 20,656 high amplitude DNA methylation sites met these criteria. As for the methylation data, we considered RNA abundance for each transcript for each sample as a function of time of death and fit cosine curves. From these fit curves, we determined the timing of peak RNA abundance (Supporting File 2). We divided genomic regions into 7 bins based on gene landmarks as above, excluding non-coding transcripts and intergenic regions, and repeated the above analyses except that rather than considering the absolute clock time of the nadir of methylation at each site, we considered the timing of the nadir of methylation relative to timing of peak RNA expression of the associated transcript. Where a DNA methylation site was associated with more than 1 transcript, the circular mean of the peak times of all associated transcripts was taken, and the timing of the nadir of methylation was taken relative to this time. There was a significant clustering of nadir methylation times relative to the timing of peak RNA abundance for DNA methylation sites in the 2 kb upstream of the transcription start site, the 1^st^ exon, the 5′UTR, and to a lesser extent the 1^st^ intron (p = 1.7×10^−42^, p = 8.5×10^−29^, p = 2.7×10^−29^, and p = 6.2×10^−13^ respectively by Rayleigh's test), with the nadir of methylation preceding the timing of peak RNA abundance by 1–3 hours for sites 2 kb upstream of the TSS, in the 5′UTR, in the 1^st^ exon, and in the 1^st^ intron (Figure 5). By contrast, no such clustering was seen for sites in other exons, other introns, and the 3′UTR (p>0.05 for all).

**Figure 5:** The timing of methylation for DNA methylation sites with high amplitude oscillations is time locked to the timing of peak RNA abundance. (A) Heat map depicting the time of the nadir of methylation relative to the timing of RNA abundance for the associated transcript, for high amplitude DNA methylation sites (i.e. amplitude of oscillation at least 10% of the mean methylation level) in or near GENCODE v14 annotated transcripts. Negative numbers mean that the nadir of methylation precedes peak RNA abundance and positive numbers indicate that the nadir of methylation follows peak RNA abundance. Red indicates a greater than expected density, while blue indicates a lesser than expected density. (B) The same data depicted as histograms in 1-hour bins. The dark line indicates the timing of peak RNA abundance. The red line indicates the angular mean time of the methylation nadir. The p-value is for Rayleigh's test for uniformity on the circle. The nadirs of methylation for sites in the 2 kb upstream of the transcription start site, the 5′UTR, the 1^st^ exon, and to a lesser extent the 1^st^ intron were significantly temporally clustered relative to the timing of peak RNA abundance (p = 8.1×10^−21^, p = 1.4×10^−15^, p = 1.2×10^−15^, and p = 3.1×10^−7^ respectively by Rayleigh's test) with the nadir of methylation preceding peak RNA abundance by 1–3 hours. There was no such temporal clustering in other exons, other introns, and the 3′UTR.

A number of clinical factors such as age [12], sex [13], [14], and presence of Alzheimer's disease [15] have been described to impact 24-hour rhythms. Moreover, dorsolateral prefrontal cortex molecular 24-hour rhythms may plausibly reflect or impact observed behavioral 24-hour rhythms. We therefore examined the impact of these factors on the amplitude and timing of 21,282 high amplitude DNA methylation sites (including intergenic sites). We assessed the effect of these variables on the parameters of DNA methylation rhythmicity by considering extended cosine models of the form M = m+(**β**_1_+**β**_2_x)*cos(t−**β**_A_−**β**_B_x) [Eq3] where x represents high vs. low age, male vs. female sex, present vs. absent Alzheimer's disease, or high vs. low behavioral rhythmicity, **β**_2_ reflects the effect of x on amplitude, and **β**_B_ reflects the effect of x on phase. Female sex, higher age, and absence of dementia were associated with an earlier average phase of rhythms of methylation (Figure 6) while the presence of Alzheimer's disease, female sex, higher age, and lower ante-mortem actigraphic rhythmicity were associated with a lower average amplitude of methylation rhythms (Figure 7).

**Figure 6:** The effects of sex, age, Alzheimer's disease, and 24-hour activity rhythms on the timing of rhythms of methylation. Circular histograms of the effect of clinical variables on the timing of the nadir of methylation of 21,282 high amplitude DNA methylation sites, in 1 hour bins. P-values determined using Rao's Test for the equality of polar directions. Dark lines indicate angular means. (A) Female vs. Male Sex. (B) Age above vs. below median (88.4 years). (C) Present vs. absent Alzheimer's Disease based on NIA-Reagan Criteria (intermediate/high = present; low/no = absent). (D) High vs. low actigraphic rhythmicity based on 24-hour activity rhythms determined ante-mortem in a subset of 134 participants by actigraphy and quantified using the interdaily stability metric as described in the text. Female sex, higher age, and absence of dementia were associated with an earlier timing of methylation nadirs.

**Figure 7:** The effects of sex, age, Alzheimer's disease, and 24-hour activity rhythms on the amplitude of rhythms of methylation. Amplitudes expressed as percentage of mean methylation at each site for 21,282 high amplitude DNA methylation sites. Horizontal lines indicate medians. Boxes indicate interquartile ranges. P-values calculated using the Wilcoxon rank-sum test. (A) Female vs. Male Sex. (B) Age above vs. below median (88.4 years). (C) Present vs. absent Alzheimer's Disease based on NIA-Reagan Criteria (intermediate/high = present; low/no = absent). (D) High vs. low actigraphic rhythmicity based on 24-hour activity rhythms determined ante-mortem in a subset of 134 participants by actigraphy and quantified using the interdaily stability metric as described in the text. Greater age, presence of AD by NIA-Reagan criteria, female sex, and lower ante-mortem actigraphic rhythmicity were associated with a lower median amplitude of cycling.

## Discussion

Using data from 420,132 DNA methylation sites spanning all 22 autosomes from 738 post-mortem human dorsolateral prefrontal cortex samples, and associated RNA sequencing data in a subset of 536 of these, this study provided evidence of 24-hour rhythms of DNA methylation whose parameters were closely related to the position of DNA methylation sites relative to gene landmarks. In particular, the timing of DNA methylation rhythms at sites proximate to transcription start sites had a characteristic phase-relationship with rhythms of RNA expression such that the nadir of methylation preceded the peak of expression by 1–3 hours. Moreover, gene regions proximate to the transcription start site were relatively enriched in DNA methylation sites with higher amplitude oscillations. In addition, higher amplitude rhythms of DNA methylation were associated with more robust ante-mortem rest-activity rhythms measured by actigraphy. Finally, age, sex, and the presence of Alzheimer's disease were significantly associated with characteristic differences in the amplitude and timing of 24-hour rhythms of DNA methylation. Taken together, these results suggest that cyclical alterations in DNA methylation status, particularly of DNA methylation sites proximate to transcription start sites, may influence 24-hour rhythms of RNA expression. Moreover, they raise the possibility that that altered 24-hour rhythms of DNA methylation may be an important mediator of the effects of age, sex, and dementia on physiological and behavioral 24-hour rhythms.

That 24-hour rhythms of histone acetylation and chromatin conformational change play an important role in driving and modulating 24-hour cycles expression of clock and clock output genes in at least some model mammalian organisms is established [3], [16], [17]. The role of DNA methylation in mammalian circadian rhythms is less clear. While DNA methylation is thought to be a relatively stable epigenetic modification, recent work has shown it to be much more dynamic than previously thought [18], [19]. A role for site-specific cycles of clock gene methylation in modulation of circadian rhythms has recently been established in Neurospora [20]. Moreover, others have recently demonstrated a role for non-circadian plasticity of DNA methylation in mediating the effect of light on the period of the intrinsic circadian clock in mice [6], and in modulating the endocrine response to changes in photoperiod in hamsters [7]. However, to our knowledge, site-specific 24-hour rhythms of DNA methylation have not to date been demonstrated in any mammalian tissue, including human neocortex. Moreover, while 24-hour rhythms of global DNA methylation have been reported in human white blood cells [21], the site-specific temporal architecture underlying this observed phenomenon was unclear, as was the extent to which similar rhythms can be found in non-blood tissues.

In this study of 420,132 CpG sites distributed across all 22 autosomes, we found evidence for significant 24-hour rhythmicity of DNA methylation in human dorsolateral prefrontal cortex with a temporal organization and amplitude exceedingly unlikely to be attributable to chance alone. Our results differ somewhat from recent studies of mouse liver [8] and suprachiasmatic nucleus [6], which found no significant 24-hour rhythms of promoter-region DNA methylation. There are several potential reasons for this discrepancy. First, there is a fundamental difference of species (human vs. mouse) and tissue (neocortex vs. liver/suprachiasmatic nucleus). Second, the present study examined methylation across the 24-hour cycle, whereas these other recent studies compared methylation levels at a small number of discrete circadian times, which would have missed rhythmic DNA methylation sites whose acrophase and nadir were out of phase with the sampling times. Third, the present study examined individual DNA methylation sites on a genome-wide scale, including all gene regions, and stratified by location relative to gene landmarks, whereas these other recent studies examined only promoter-region DNA methylation sites. Finally, the present study had a much larger number of tissue samples (n = 738), allowing greater statistical power to detect rhythmicity.

 Our data support a differential functional role for 24-hour rhythms of DNA methylation depending on the location of the DNA methylation site. Regions proximate to transcription start sites (e.g. within 2 kb upstream of the transcription start site, the 5′UTR, the 1^st^ exon, or the 1^st^ intron) were particularly highly enriched for high amplitude rhythmic DNA methylation sites, and the timing of methylation rhythms at these sites was time-locked to rhythms of local gene expression, with the timing of the nadir of methylation preceding the peak of gene expression by 1–3 hours. This suggests that 24-hour rhythms of DNA methylation at sites proximate to transcription start sites may play a particular role in regulating the transcription of rhythmic transcripts. This is in keeping with the hypothesis that methylation sites near the transcription start site are most likely to play a role in regulating transcription, while those elsewhere may play non-transcription related roles [22]. Meanwhile, the clustering of methylation nadir times between 18:00 and 22:00 for sites removed from transcription start sites is in concordance with previous work in mouse liver showing a global decrease in DNA methylation in the later afternoon [23].

In this study, men had relatively later rhythms of DNA methylation than women. This is in keeping with our previous work showing that men have 24-hour rhythms of neocortical clock gene expression [24] and activity [25] that are relatively delayed compared to females. We also observed in our data that greater age was associated with relatively earlier and lower amplitude rhythms of DNA methylation and that the presence of pathologically confirmed Alzheimer's disease was also associated with relatively lower amplitude and delayed rhythms of rhythms of DNA methylation. This is concordant with previous work showing a relative phase advance of several measures of circadian rhythmicity with increasing age [25] [12], and a relative decrease in amplitude of other measures of circadian rhythmicity in the context of dementia [15], [26]. Finally, in the subset of 134 individuals who had actigraphic recordings prior to death, those individuals who had less robust 24-hour rhythmicity on their actigraphic recordings also had on average somewhat attenuated rhythms of DNA methylation at the time of death, supporting a link between 24-hour rhythms of neocortical DNA methylation, and 24-hour rhythms of behavior. As this study was cross-sectional in nature, the causal relationship between age, dementia, dorsolateral prefrontal cortex 24-hour DNA methylation rhythms, and behavioral 24-hour rhythms cannot be determined from these data alone, and further studies, particularly in animal models of aging and neurodegeneration, will be needed. Moreover, whether these differences are fundamentally due to differences a the level of the dorsolateral prefrontal cortex, or reflect differences in the function of the central circadian pacemaker, or even differences in confounding environmental exposures cannot be deduced from our data.

This study has a number of methodological strengths. We assessed DNA methylation and RNA expression on a genome-wide scale and in all gene regions, allowing comparison of the circadian properties of DNA methylation sites in the promoter region, 5′UTR, exons, introns, 3′UTR, and intergenic regions. Moreover, we measured DNA methylation and RNA expression from the same samples, allowing the inference of temporal correlations. Also, the large number of subjects and high temporal density of sampling (>50 data points per hour) allows a much more precise consideration of phase relationships than would be possible in an experiment where the data were sampled less frequently (e.g. every hour or two) as is the case in many circadian studies. Moreover, the use of neocortical tissue from humans rather than model organisms enhances the potential for clinical translation. In addition, the fact that all of the participants were organ donors ensures accurate determination of time of death and short postmortem intervals. Finally, these data were obtained from subjects living in the community, rather than in a laboratory, making the data more directly applicable to real-world scenarios.

In considering these data, a few methodological points are worth noting. In this study, we inferred group-level average 24-hour rhythms of DNA methylation and RNA expression from postmortem samples and were limited in exploring individual level differences in 24-hour rhythmicity. However, ethical factors preclude serial sampling of neocortical tissue from naturally behaving individuals, which would be necessary to obtain true individual-level characterization of 24-hour rhythms of neocortical DNA methylation. Moreover, behavioral state at death (e.g. sleep/wake) and environment (e.g. light exposure) at death were not known. Therefore, it is possible that the observed 24-hour rhythms were confounded by rhythmic differences in behavior, environment, behavioral state, or medical status at death. While laboratory-based experimental designs (e.g. forced-desynchrony experiments) exist that can decouple environmental/behavioral effects from circadian effects, similar studies on human neocortical tissue cannot be performed in the context of such experiments. Further studies of neocortical DNA methylation in model organisms studied under controlled conditions will be needed to distinguish environmental, behavioral, and circadian components of 24-hour rhythms of neocortical DNA methylation. Finally, DNA methylation was assessed using data from a beadset (the Illumina 450k Array) with specifically selected methylation sites rather than a more unbiased approach that generates truly genome-wide data. Thus, it is conceivable that the methylation sites represented on the beadset platform that we used may not be completely representative of DNA methylation sites as a whole, particularly with regard to intergenic regions that are relatively under-represented on the Illumina 450k Array.

Taken together, the data from this study suggest that as in *Neurospora*, 24-hour cycles of DNA methylation, particularly at sites proximate to the transcription start site, may be an important mechanism regulating 24-hour rhythms of gene expression in the human brain and potentially other human and mammalian tissues. Furthermore, they add to the growing body of evidence that mammalian DNA methylation, once thought to be a relatively stable epigenetic mark, can be dynamic on time scales as short as hours. These results also invite examination of the role of 24-hour rhythms of DNA methylation in the regulation of 24-hour rhythms of gene expression and tissue biology in other clinically important human tissues such as myocardium and liver. Moreover, work in mammalian model systems is needed to identify mechanisms underlying site-specific 24-hour rhythmic DNA methylation.

## Materials and Methods

### Participants

 This study included participants from two ongoing longitudinal cohort studies of older individuals: the Religious Orders Study (ROS) and the Rush Memory and Aging Project (MAP). The MAP is a community-based study of aging in the greater Chicago area. Recruitment and assessment procedures are described elsewhere [27]. Participants are free of dementia at study enrollment, and agree to annual evaluations and brain donation upon death. At the time of the current analyses, 1667 individuals had completed baseline evaluation and 485 had died, with cerebral cortex DNA methylation data passing quality control criteria (see below) available from 402. The ROS is a longitudinal study of aging in Catholic priests, nuns, and brothers from across the USA. A detailed description can be found elsewhere [28]. At the time of the current analyses, 1172 ROS participants had completed baseline evaluation and 569 had died, with cerebral cortex DNA methylation data passing quality control criteria (see below) available from 346. Of the 748 samples with adequate DNA methylation data, 2 did not have an accurate time of death recorded and were excluded from our analyses. Because all participants in the ROS and MAP are organ donors, time of death is well captured in both cohorts. After quality control filtering (see below) data from 738 participants were included in the current analyses. Characteristics of the study participants are shown in Table 1.

### Statement of ethics approval

The study was conducted in accordance with the latest version of the Declaration of Helsinki and was approved by the Institutional Review Board of Rush University Medical Center. Written informed consent was obtained from all subjects, followed by an Anatomic Gift Act for organ donation.

### Evaluation of dorsolateral prefrontal cortex DNA methylation

DNA methylation was assessed in 746 human postmortem dorsolateral prefrontal cortex samples as previously described [29], [30]. Frozen 100 mg dorsolateral prefrontal cortical blocks were thawed on ice and gray matter was manually dissected for DNA extraction using the QIAamp DNA Mini Kit (Qiagen, Venlo, Netherlands; Cat: 51306). DNA concentration was measured by using the Quant-iT PicoGreen Kit (Life Technologies, Carlsbad, CA) and 16 µL of DNA from each sample at a concentration of 50 ng/µL was assayed using the Illumina Infinium HumanMethylation450k Bead Chip assay (Illumina, San Diego, CA) by the Broad Institute's Genomics Platform. Raw data generated from Illumina 450k platform were processed using Genome Studio software Methylation Module v1.8 (Illumina, San Diego, CA) to generate beta-values and detection p-values for 485,513 CpG across the human genome following color channel normalization and background removal. We excluded from analysis probes with detection p-values>0.01 in any sample, probes in which 47/50 nucleotides matched sex chromosome sequences during sequence alignment using BLAT [31], probes in which a SNP with a minor allele frequency> = 0.01 exists within 10 base pairs upstream or downstream of the CpG site, and probes on the sex chromosomes, leaving 420,132 autosomal CpGs in the dataset.

Sample quality was assessed using principal component analysis and we included only those samples having principal component 1, 2 and 3 (PC1, PC2 and PC3) values within +/−3 standard deviations from their respective means. We also excluded subjects with poor bisulfite conversion efficiency, defined as having at least 2 of the 10 bisulfite conversion control probes failing to reach a value of 0.8. After these exclusions, we had 738 remaining samples.

Missing data were imputed and approximated using the k-nearest neighbor algorithm with k = 100. Following quality control filtering as above, data from 738 subjects were available for analysis.

### Evaluation of clock gene transcript expression

RNA was extracted from dorsolateral prefrontal cortex blocks from a subset of 536 individuals (Table S1) using the miRNeasy mini kit (Qiagen, Venlo, Netherlands) and the RNase free DNase Set (Qiagen, Venlo, Netherlands). These samples were quantified by Nanodrop (Thermo Fisher Scientific, Waltham, MA) and an Agilent Bioanalyzer was used to assess quality. Samples with Bioanalyzer RNA integrity (RIN) score of 5 or less or with less than 5 µg of RNA were excluded. RNA sequencing library preparation was performed by the Broad Institute Genomics Platform using the strand specific dUTP method [32] with poly-A selection [33]. This consists of poly-A selection followed by first strand specific cDNA synthesis, and then uses dUTP for second strand specific cDNA synthesis followed by fragmentation and Illumina adapter ligation for library construction. Sequencing was performed on the Illumina HiSeq with 101 bp paired-end reads and achieved coverage of 150M reads for the first 12 samples, which served as a deep coverage reference. The remaining samples were sequenced with coverage of 50M reads. Next, we trimmed off beginning and ending low quality bases, trimmed adapter sequences from the reads, and removed ribosomal RNA reads. We then used the Bowtie 1 software package [34] to align the trimmed reads to the reference genome. Finally, we used the RSEM software package to estimate, in units of fragments per kilobase per million fragments mapped (FPKM), expression levels for 69,605 GENCODE v14 transcripts overlapping with high amplitude DNA methylation sites or whose transcription start sites were within 2 kb of such DNA methylation sites.

### Assessment of clinical covariates

Age was computed from the self-reported date of birth and the date of death. Sex was recorded at the time of the baseline interview.

Individuals were classified as having/not having clinical dementia as previously described [35]. Briefly, trained technicians annually administered 21 cognitive tests spanning 5 cognitive domains [36]. The results of cognitive tests were reviewed by a neuropsychologist to determine the presence or absence of cognitive impairment. At each annual evaluation, a clinician combined the most current available cognitive and clinical data to determine whether the subject had dementia or not according to the NINDS-ADRDA criteria [37]. The final determination of the presence/absence of dementia at the time of death was based on consideration of all cognitive assessments prior to death. For a pathological diagnosis of Alzheimer's disease, as described previously [38], Bielschowsky silver stain was used to visualize neurofibrillary tangles, diffuse plaques, and neuritic plaques in the frontal, temporal, parietal, and entorhinal cortices, and the hippocampus. Braak stages 0 through VI were assigned based upon the distribution and severity of neurofibrillary tangle pathology [39]. All cases received a neuropathologic diagnosis of no Alzheimer's disease, low likelihood Alzheimer's disease, intermediate likelihood Alzheimer's disease, or high likelihood Alzheimer's disease based on the National Institutes of Aging (NIA)-Reagan criteria [40].

A subset of 134 participants in the MAP cohort had undergone up to 10 days of actigraphy a median of 16.0 months prior to death (Table S2). Study staff placed actigraphs (Actical, Philips Respironics, Bend, OR) set to record in 15-second epochs on participants' nondominant wrists for up to 10 days. We calculated the interdaily stability statistic [26], [41], which is a measure of the day-to-day regularity of the rest-activity rhythm with 1 indicating perfect regularity, and 0 indicating no regularity.

### Analysis

For both the DNA methylation and RNA expression data, prior to further analyses, we sought to account for the contribution of identifiable biological (age, sex, presence/absence of clinical dementia) and technical (source cohort, post-mortem interval, batch) factors to the overall variance in expression or methylation levels at each site, and thereby decrease the “noise” in the data, by regressing the methylation and expression data against these factors. After fitting the model, the residuals of the model were kept and represent the expression or methylation level at each site adjusted for these factors. This accounts for the contribution of these factors to the overall “noise” in the mean expression or methylation levels at each site, but does not preclude assessment of the effects of these factors on the amplitude and phase of rhythmicity. Finally, we scaled the methylation or expression level at each site to the standard deviation for that site considering all 738 subjects.

To identify temporal patterns in DNA methylation at each CpG site, we considered DNA methylation as a function of clock time of death, with each subject contributing a single data point to a time series spanning 24-hours. First, to visually identify trends, we divided the data into 4-hour bins and plotted the mean expression levels and 95% confidence intervals of the means. Visual inspection of these figures suggested that 24-hour rhythms of DNA would be appropriately modeled using cosine curves. Therefore, we parameterized daily variation in the DNA methylation data using functions of the form: M = m+(**β**_1_)*cos(t−**β**_A_)..[Eq1] where m is the mesor (the mean value considering all time points), (**β**1) is the amplitude of oscillation, **β**_A_ is the timing of the peak, and t is the time of death. For computational efficiency, equivalent linearized models of the form M = m+**β**_c_*cos(t)+**β**_s_*sin(t).[Eq2] were fit using the R function lm() and the parameters **β**_1_ and **β**_A_ from Eq1 were calculated using the formulae **β**_1_ = (**β**_c_^2^+**β**_s_^2^)^0.5^ and **β**_A_ = arctan(**β**_s_/**β**_c_). For all our analyses, we fixed the period at 24-hours. This is a limitation of any study design where each individual contributes only 1 data point to a 24-hour sampling period. All clock times were converted to radians (2π radians = 24 hours; 0 radians = midnight) for analysis and then converted back to hours for the purposes of visual representation.

In our primary analyses, we examined all 420,132 sites together, to identify aggregate patterns of rhythmicity. To quantify the probability that the observed data could have occurred by chance alone, we performed a series of analyses comparing the observed data to 10,000 permuted null datasets generated by randomly shuffling the times of death in our data while preserving the correlation between DNA methylation sites. For each DNA methylation site in each of these permuted null datasets, we fit a cosine curve as above, calculated the proportion of variance at that site explained by the cosine curve, and determined the time of the acrophase (**β**_A_) and nadir (**β**_A_-**π**) of the fit curve. We then carried out four analyses comparing the observed to the permuted null data: 1) we calculated the mean total proportion of variance collectively explained by the individually fit cosine curves in each of the 10,000 permuted null datasets and in the observed data, and determined the proportion of null datasets in which this was as large or larger than the observed data. 2) We repeated this for the median total proportion of variance collectively explained by the individually fit cosine curves. 3) We generated a sorted mean empiric null distribution of proportions of variance explained by taking the mean of the 10,000 sorted permuted null distributions (each of length 420,132), and used the Wilcoxon signed-rank test to compare this with the observed distribution of 420,132 proportions of variance explained. 4) We used the Rao test [42] to compare the observed distribution of methylation nadir times (**β**_A_-**π**) to those in the 10,000 permuted null datasets.

We next examined the relationship between the estimated parameters of rhythmicity (amplitude and phase) at each DNA methylation site, and the location of the site relative to nearby transcription start sites. First, we focused in on regions of the genome within 20 kb of GENCODE v14 annotated transcription start sites [43]. We divided these regions into 80 equally-spaced 500 bp bins from −20 kb to +20 kb relative to transcription start sites such that, for instance, the −20,000 bp to −19,500 bp bin contained all genomic regions ranging from −20,000 bp to −19,500 bp of any GENCODE-annotated transcription start site. We identified DNA methylation sites contained in each bin, determined the probability distribution of the timing of the methylation nadirs at these sites, and represented this visually as a heat map with the 24-hour cycle divided into 24 equal 1-hour windows. Visual inspection of this heat map suggested a differential phase distribution of DNA methylation sites within 1 kb of transcription start sites, those more than 1 kb upstream of transcription start sites, and those more than 1 kb downstream of transcription start sites. Therefore, we grouped these DNA methylation sites into one of three groups (−20 kb to −1 kb, −1 kb to +1 kb, and +1 kb to +20 kb), plotted the distribution of the timing of the methylation nadirs in each group as a histogram, and compared these temporal distributions using Rao's test [42].

We then went on to examine for associations between physical position and the amplitude of 24-hour cycling. We classified individual DNA methylation sites as high amplitude the peak-to-trough amplitude of rhythmicity was greater than 10% of the mean value of methylation at that site. Using the same bins relative to transcription start sites as above, we determined the proportion of DNA methylation sites that are high amplitude sites, as a function of position from the nearest transcription start site. Enrichment was tested using the chi-square test.

We then repeated the above analyses, except that rather than dividing the genome into bins based on position relative to transcription start sites, we incorporated information about other gene landmarks and divided genomic segments into 9 bins: regions within 2 kb upstream of transcription start sites, in the 5′UTR, in the 1^st^ exon, in the 1^st^ intron, in other exons, in other introns, and in the 3′UTR of protein coding transcripts; regions in or within 2 kb upstream of non-protein coding transcripts, and intergenic regions (defined as all other genomic regions).

Following this, we examined the relationship between rhythms of DNA methylation and RNA abundance for 20,656 DNA methylation sites classified as high amplitude cycling sites (based on an amplitude of cycling >10% of the mean value of methylation) and lying in or within 2 kb of GENCODE v14 annotated transcripts in a subset of 536 subjects who had both DNA methylation and RNA sequencing data. We considered all GENCODE v14 [43] isoforms detected in at least 10% of our samples. We divided genomic regions into 7 bins based on gene landmarks as above, excluding non-coding transcripts and intergenic regions, and repeated the above analyses except that rather than considering the absolute clock time of the nadir of methylation at each site, we considered the timing of the nadir of methylation relative to timing of peak RNA expression of the associated transcript. Where a particular DNA methylation sites was associated with more than one transcript, the angular mean of the peak time of all associated transcripts was taken, and the timing of the nadir of methylation was taken relative to this time. These analyses were first visually represented as a heat map, and then a formal bin-by-bin analysis was performed using Rayleigh's test [44] to test for temporal clustering of methylation nadir times relative to the timing of peak RNA expression.

We next examined the impact of age, sex, presence/absence of Alzheimer's disease, and the regularity of ante-mortem rest-activity rhythms measured by actigraphy on the amplitude and timing of 21,282 high-amplitude DNA methylation (those described above plus high amplitude intergenic sites). We dichotomized age into high vs. low based on the median (i.e. above or below 88.4 years age time of death), sex into male vs. female, and Alzheimer's disease into present/absent based on NIA-Reagan criteria [40] intermediate/high vs. low/no. We dichotomized the subset of 134 individuals who had antemortem actigraphy into high vs. low behavioral rhythmicity based on their interdaily stability values being above or below the median (i.e. above or below 0.49). At each high amplitude rhythmic DNA methylation site, we fit extended cosine models of the form M = m+(**β**_1_+**β**_2_x)*cos(t−**β**_A_−**β**_B_x) [Eq3] where x represents high vs. low age, male vs. female sex, present vs. absent Alzehimer's disease, or high vs. low behavioral rhythmicity, **β**_2_ reflects the effect of x on amplitude, and **β**_B_ reflects the effect of x on phase. As above, for computational efficiency, we fit linearized versions of Eq3 similar to Eq2 using the function lm() and determined the values of **β**_2_ and **β**_B_ from this. We then used the Wilcoxon rank-sum test to compare the distribution of amplitudes between levels of each dichotomous predictor, and used Rao's test to compare the distribution of methylation nadir times between levels of each dichotomous predictor.

In total, the analyses described above include 24 independent hypotheses tested. Applying the Bonferroni-Holm correction we therefore set the threshold for significance for each of these tests at p = 0.05/24 = 0.002.

For all analyses, visual examination of residual plots confirmed that cosine curves of the form described above provided a functionally appropriate description of temporal trends and confirmed model assumptions of homogeneous variance.

## Supporting Information

Table S1 Clinical characteristics of the subjects with and without RNA expression data.
(DOC)

Table S2 Clinical characteristics of the subjects with and without ante-mortem actigraphy data.
(DOC)

File S1 Parameters of cosine curves at all 420,135 CpG sites.
(ZIP)

File S2 Parameters of cosine curves for 69,605 GENCODE v14 transcripts containing or within 2 kb of high amplitude CpG sites.
(ZIP)
